The article "Chalcone 9X Contributed to Repressing Glioma Cell Growth and Migration and Inducing Cell Apoptosis by Reducing FOXM1 Expression In Vitro and Repressing Tumor Growth In Vivo" was published in 2022. Journal: Biomed Res Int.

# Chalcone 9X Contributed to Repressing Glioma Cell Growth and Migration and Inducing Cell Apoptosis by Reducing FOXM1 Expression In Vitro and Repressing Tumor Growth In Vivo

**DOI:** 10.1155/2022/8638085

**Published:** 2022-08-08

**Authors:** Chenguang Li, Rui Wang, Wenshi Guo, Xu Feng, Ning Guan

**Affiliations:** Department of Neurosurgery, The First Affiliated Hospital of Jinzhou Medical University, Jinzhou 121001, China

## Abstract

**Objective:**

Natural and synthetic chalcones played roles in inflammation and cancers. Chalcone 9X was an aromatic ketone that was found to inhibit cell growth of hepatic cancer and lung cancer cells. In this study, we wanted to investigate the functions of Chalcone 9X in glioma.

**Materials and Methods:**

Chemical Chalcone 9X was added in human glioma cell lines (U87 and T98G cells) and normal astrocyte cell lines (HA1800) with various concentrations (0 *μ*mol/L, 20 *μ*mol/L, 50 *μ*mol/L, and 100 *μ*mol/L). CCK-8 assay was used to measure cell viability. Flow cytometric assay was used to measure cell apoptotic rates. Wound healing assay and transwell assay were used to measure cell invasion. RT-PCR was used to detect relative mRNA expressions, and the protein expressions were detected by western blot (WB) and immunohistochemical staining (IHC). Finally, nude mouse xenograft assay was performed to prove the effects of Chalcone 9X in vivo.

**Results:**

Results revealed that Chalcone 9X treatment suppressed cell viability and cell migration capacity; it could also induce cell apoptosis in U87 and T98G cells with dose dependence. However, it had little cytotoxicity to normal astrocyte HA1800 cells. Moreover, Chalcone 9X treatment could repress the mRNA and protein expressions of FOXM1 in human glioma cell lines, which was an oncogene that could promote the progression and malignancy of glioma. In addition, FOXM1 overexpression dismissed the Chalcone 9X effects on cell proliferation, apoptosis, and migration in human glioma cell lines. Finally, in vivo assay showed that Chalcone 9X treatment repressed the expression of FOXM1, which inhibited the tumor growth of a xenograft model injected with U87 in nude mice.

**Conclusions:**

In all, we found that Chalcone 9X could suppress cell proliferation and migration and induce cell apoptosis in human glioma cells, while it has little cytotoxicity to normal astrocyte cells. Therefore, we uncovered a novel way that Chalcone 9X could inhibit FOXM1 expression and repress the progression and biofunctions of glioma cells, which might be a potential therapeutic drug for treating human glioma.

## 1. Introduction

Glioma is a king of prevalent cancer on central nervous system worldwide [1–4], and it is divided into astrocytoma, oligodendroglioma, and ependymal tumor [1]. Researchers reported that its incidence has been obviously increased for the past 20 years [1, 3]. Because of its variability, no specific treatments and strategies have been developed and applied [5, 6]. Therefore, it is urgent to find some new effective therapies and drugs with significant effects and low cytotoxicity to hinder the development of glioma.

The article "Chalcone 9X Contributed to Repressing Glioma Cell Growth and Migration and Inducing Cell Apoptosis by Reducing FOXM1 Expression In Vitro and Repressing Tumor Growth In Vivo" was published in 2022. Journal: Biomed Res Int.

Natural and chemical synthetic chalcones have been revealed to play critical roles in some biological functions, such as inflammation [7–9] and antibacterial effects [10, 11]. Furthermore, more studies demonstrated that chalcones could inhibit tumor progression in various cancers [12–19], including glioma [15, 18]. For example, Mendanha et al. found that Chalcone 1 could induce cell apoptosis of glioblastoma (GBM), which was triggered by the cell cycle arrest in the G2/M checkpoint, and might be a potential to provide a new treatment alternative for GBM^15^. Moreover, Wang et al. also discovered that flavokawain B (FKB), a natural kava chalcone, induced protective autophagy signaling pathway in GBM cells, which indicated that the combination treatment of FKB with autophagy inhibitors might be an effective strategy for GBM^18^.

The chemical synthetic chalcone 4′-hydroxyl-3,4-dimethoxyl-3′-methoxylchalcone (Chalcone 9X) was an aromatic ketone that had been demonstrated to have some antitumor activities in human lung cancer cells and hepatic cancer cells [19]. Researches revealed that Chalcone 9X could induce cell apoptosis and inhibit invasion and migration capacities through activating Caspase-3 and Caspase-8 signaling pathways in lung cancer cells and hepatic cancer cells in vitro and in vivo [19]. However, the functions of Chalcone 9X in other tumors remained unknown, and whether Chalcone 9X could affect glioma cells remained unclear.

In this study, we wanted to investigate whether Chalcone 9X played some roles in glioma. Our preliminary results hinted that it showed some antitumor activities in human glioma cells. As a result, we explored the potential molecular mechanism of Chalcone 9X in glioma in vitro and in vivo.

## 2. Materials and Methods

### 2.1. Chalcone 9X Synthesis

The chemical Chalcone 9X was synthesized with the standard Claisen-Schmidt aldol condensation protocols from El-Mahdy et al. [20] and Konoike et al. [21] The 3,4-dimethoxyl benzaldehyde was added into a stirred solution of 4-hydroxyl-3-methoxylacetophenone, and the solution was added with NaOH and ethanol. The synthetic reaction was finished at room temperature for 48 h, which was then quenched in ice-cold water and acidized with 18% HCl. The separated product was filtered. Finally, the crude product was recrystallized from ethanol and stored until usage. The chemical formula of Chalcone 9X is C_18_H_18_O_5_, and the molecular weight is 314 g/mol. Chalcone 9X was diluted into concentrations of 20 *μ*mol/L, 50 *μ*mol/L, and 100 *μ*mol/L to treat cells.

The article "Chalcone 9X Contributed to Repressing Glioma Cell Growth and Migration and Inducing Cell Apoptosis by Reducing FOXM1 Expression In Vitro and Repressing Tumor Growth In Vivo" was published in 2022. Journal: Biomed Res Int.

### 2.2. Cell Culture

Human normal astrocyte cell line HA1800 and human glioma cell lines (U87, T98G) were obtained from American Type Culture Collection (ATCC; Manassas, VA, USA), and cells were cultured in DMEM (Hyclone, Massachusetts, USA) with 10% fetal bovine serum (FBS; Gibco, Grand Island, NY, USA), 100 U/mL penicillin (Hyclone, South Logan, UT, USA), and 100 U/mL streptomycin (Hyclone, South Logan, UT, USA). Cells were cultivated in an atmosphere with 37°C and 5% CO2.

### 2.3. Construction of Plasmid and Cell Transfection

The full length of human FOXM1 cDNA was synthesized and constructed into a pCDNA3.1 (Invitrogen, Carlsbad, CA, USA) vector, resulting in FOXM1-pcDNA for its overexpression, which was named p-FOXM1. And scrambled oligonucleotides were synthesized to be used as the negative control, which was named p-NC. U87 and T98G cells were preincubated on six-well plates to about 50% confluence, which was then transfected by incubation with p-FOXM1 or p-NC with Lipofectamine 2000 (Invitrogen, Carlsbad, CA, USA) according to the manufacturer's protocol. U87 and T98G cells with FOXM1 stable overexpression were obtained. Then, Chalcone 9X was used to treat these prepared cells, and cells were harvested after 48 h for further analysis.

### 2.4. CCK-8 Assay

Cell viability of human normal astrocyte cell line HA1800 and glioma cells (U87 and T98G) were detected by a cell counting kit-8 (CCK-8) assay (Dojindo, Rockville, Japan). Cells were seeded on 96-well plates (2 × 10^3^ cells/mL) and cultivated in an incubator. Then, 10 *μ*L CCK-8 agent was added to the prepared cells at 24 h, 48 h, and 72 h. Finally, the absorbance of each well was measured at 450 nm using a microplate reader (Thermo Fisher, USA). Three independent experiments were repeated to get the mean value.

### 2.5. Flow Cytometric Analysis

Cell apoptotic rates were measured by flow cytometric analysis. After Chalcone 9X treatment for the indicated time, prepared glioma cells were washed with PBS three times and digested with 0.25% trypsin. Then cells were stained with FITC-Annexin V and Propidium iodide (PI) solution with 50 *μ*g/mL at room temperature for 30 min. At last, stained cells were subjected to a FACScan Calibur flow cytometer (BD Biosciences Becton-Dickinson, Franklin Lakes, USA) to calculate apoptotic cell rates.

### 2.6. Transwell Assay

Cell migration ability was measured by Transwell assay. U87 and T98G cells (5 × 10^4^ cells/well) were plated to the top of upper chambers (Corning, NY, USA) on the noncoated membranes with a 200 *μ*L serum-free medium. The lower chambers were added with 500 *μ*L 10% FBS and DMEM (Hyclone, Massachusetts, USA). After 24 h, the cells that remained in the upper chambers were removed; however, migrated cells through the membranes were stained with 95% methanol for 15 min and then stained with 0.1% crystal violet for 20 min. Finally, the migrated cells were counted and examined under a light microscope (Olympus, Tokyo, Japan).

The article "Chalcone 9X Contributed to Repressing Glioma Cell Growth and Migration and Inducing Cell Apoptosis by Reducing FOXM1 Expression In Vitro and Repressing Tumor Growth In Vivo" was published in 2022. Journal: Biomed Res Int.

### 2.7. Wound Healing Assay

Wound healing assay was used to measure glioma cell migration ability. U87 and T98G cells were cultured in 60-mm tissue culture plates for 24 h. Then a pipette tip was used to create an artificial wound, and the wells were washed with PBS three times to remove the detached cells. Furthermore, U87 and T98G cells were treated with Chalcone 9X (0 *μ*mol/L, 20 *μ*mol/L, 50 *μ*mol/L, and 100 *μ*mol/L) in new media for 48 h. The wounds were photographed and measured using an inverted microscope (Leica, Germany).

### 2.8. RNA Extraction and RT-PCR

Total RNAs were extracted by using a TRIZOL Reagent (Invitrogen, CA, USA) from cells following the manufacturer's protocol. Then, the cDNA was reversed by using a PrimeScript™ RT reagent Kit (Takara, Tokyo, Japan) according to the manufacturer's protocol. PCR primers were synthesized by RiboBio Co., Ltd. (Guangzhou, China). Primer sequences were listed as follows: FOXM1—forward: 5′-CACTTGGATTGAGG ACCACTT-3′, reverse: 5′-GTCGTTTCTGCTGTGATTCC-3′; GAPDH—forward: 5′-GGAGTCCACTGGTGTCTTCA-3′, reverse: 5′-GGGAACTGAGCAATTGGTGG-3′. SYBR Premix Ex Taq II (Takara, Tokyo, Japan) was used to detect relative mRNA expressions according to the manufacturer's protocol; the 2^-△△CT^ method was used to calculate expressions, which were normalized to GAPDH.

### 2.9. Protein Extraction and Western Blot

Total proteins were extracted from U87 and T98G cells using a RIPA buffer (Beyotime, Shanghai, China) with a phosphatase inhibitor (Beyotime, Shanghai, China) on the ice. The proteins were extracted from tumor tissues for each animal in each group. Then, protein concentrations were measured by using a BCA Protein Assay (Beyotime, Shanghai, China). 50 *μ*g total protein was added onto 10% SDS-PAGE for electrophoresis, and the separated proteins were transferred onto PVDF membranes. Membranes were blocked with 5% nonfatty milk at room temperature for 2 h and washed by Tris-buffered saline with Tween (TBST) for three times, which were then incubated with primary antibodies overnight at 4°C. All primary antibodies were purchased from Abcam (Abcam, Cambridge, USA), including Wnt (ab28472, 1 : 1000, 39 kDa), *β*-catenin (ab32572, 1 : 5000, 92 kDa), p-*β*-catenin (ab81305, 1 : 10000, 70 kDa), ERK1 (ab32537, 1 : 1000, 44, 42 kDa), p-ERK1 (ab201015, 1 : 1000, 44, 42 kDa), GSK3*β* (ab32391, 1 : 5000, 46 kDa), p-GSK3*β* (ab68476, 1 : 2000, 47 kDa), FOXM1 (ab207298, 1 : 1000, 84 kDa), Vimentin (ab8978, 1 : 1000, 57 kDa), N-cadherin (ab76057, 1 : 1000, 100 kDa), E-cadherin (ab40772, 1 : 5000, 97 kDa), and GAPDH (ab8245, 1 : 5000, 36 kDa). Then, membranes were incubated with matched secondary antibodies (1 : 5000, Abcam, Cambridge, USA) for 1 h. Protein bands were visualized by Odyssey Infrared Imaging System (LI-COR, Lincoln, NE, USA).

The article "Chalcone 9X Contributed to Repressing Glioma Cell Growth and Migration and Inducing Cell Apoptosis by Reducing FOXM1 Expression In Vitro and Repressing Tumor Growth In Vivo" was published in 2022. Journal: Biomed Res Int.

### 2.10. Tumor Xenograft in Nude Mice

Eighteen nude male BALB/c mice were included (SLAC Laboratory Animal, Shanghai, China), which were 4 weeks old and weigh 15-20 g. Mice were raised in standard laboratory conditions and fed food and water. Then, the nude mice were injected with U87 cells (5 × 10^6^ cells in 0.1 mL of PBS) on the right flanks. After two weeks, these mice were divided into three groups (*n* = 6), including the model group, Chalcone 9X 20 mg/kg group, and Chalcone 9X 40 mg/kg group. Chalcone 9X was provided by tail vein injection once a day for four weeks, and tumor volumes of nude mice in three groups were observed every week. The tumor volumes were calculated with *V* = *π*/6 × length × width × height. Mice were sacrificed; tumor tissues were obtained for further research. The extracted tumors were frozen with optimal cutting temperature (OCT) compound (Sigma-Aldrich; Merck KgaA, USA) at −20°C, which were then stored at −80°C until use. All procedures were carried out according to the Guide for the Care and Use of Laboratory Animals of the National Institutes of Health. This study was approved by the Animal Care Ethics Committee of our hospital.

### 2.11. Immunohistochemical Staining

The extracted tumor tissues were sliced at a thickness of 10 *μ*m and were placed on gelatin-coated glass slides. Furthermore, the sliced tumor tissues were fixed with 4% paraformaldehyde (PFA) for 15 min, which were incubated with methanol containing 3% hydrogen peroxide for another 20 min. The sliced tumor tissues were placed with 0.3% Triton X-100 in PBS for 20 min. Besides, the tissues were blocked with the blocking solution for 1 h, which was fixed with 0.1% BSA (Sigma-Aldrich; Merck KgaA, USA), 0.3% Triton X-100, and 1.5% FBS (Hyclone; Cytiva, USA). Then, the tissues were incubated with the primary antibodies overnight at 4°C, including FOXM1 (ab207298, Abcam, Cambridge, USA) and Caspase-3 (ab13847, Abcam, Cambridge, USA). Finally, the incubated tissues were subsequently washed with PBS two times and then incubated with biotinylated anti-rabbit (cat. no. BA-1000), and anti-rat (cat. no. BA-4000) IgG (H+L) antibodies (1 : 400, Abcam, Cambridge, MA, USA) were labeled secondary antibodies. The tumor tissues were sealed and observed under an inverted microscope (IX73, Olympus, Tokyo, Japan). To determine cell proliferation of tumor tissues, four high-powered fields of vision were obtained from each group. The average number of FOXM1+ cells or Caspase-3+ cells was used for statistical analysis, which was quantified as the protein expression.

The article "Chalcone 9X Contributed to Repressing Glioma Cell Growth and Migration and Inducing Cell Apoptosis by Reducing FOXM1 Expression In Vitro and Repressing Tumor Growth In Vivo" was published in 2022. Journal: Biomed Res Int.

### 2.12. Statistical Analysis

The data were analyzed by SPSS 18.0 (Chicago, IL, USA) and GraphPad Prism 5.0 (La Jolla, CA, USA). Data were analyzed according to three independent experiments. Statistical significance between groups were analyzed by the SNK method followed by one-way ANOVA. *p* < 0.05 was considered to be a statistically significant difference.

## 3. Results

### 3.1. Chalcone 9X Suppressed Cell Proliferation in U87 and T98G Cells

We wanted to explore the functions of Chalcone 9X in glioma and whether it had cytotoxicity in normal cells. Chalcone 9X with concentrations of 0 *μ*mol/L, 20 *μ*mol/L, 50 *μ*mol/L, and 100 *μ*mol/L were used to treat human glioma cell lines (U87 and T98G) and HA1800 for 24 h, 48 h, and 72 h. Then, cell viability was measured by CCK-8 assay. Results showed that Chalcone 9X treatment significantly repressed the cell viability of U87 and T98G cells in a dose-dependent manner at the time of 48 h and 72 h (Figures 1(a)–1(f)) (*p* < 0.05). Importantly, Chalcone 9X treatment had little influence on cell viability for HA1800 cells after 24 h, 48 h, and 72 h (Figures 1(g)–1(i)) (*p* > 0.05), which indicated that Chalcone 9X had little cytotoxicity to HA1800 cells. These results indicated that Chalcone 9X suppressed cell proliferation in U87 and T98G cells, while it had little cytotoxicity on human normal astrocyte HA1800 cells.

### 3.2. Chalcone 9X Induced Cell Apoptosis in U87 and T98G Cells

To investigate whether Chalcone 9X could affect cell apoptosis in glioma cells, Chalcone 9X was treated in human U87 and T98G for 48 h. Then, cell apoptosis was measured by FACS assay. Results showed that cell apoptotic rates of glioma cells treated with Chalcone 9X were markedly higher than the control group in a dose-dependent manner after 48 h (Figures 2(a)–2(d)) (*p* < 0.05), which indicated that Chalcone 9X treatment significantly induced cell apoptosis and repressed cell proliferation in U87 and T98G cells.

### 3.3. Chalcone 9X Repressed Cell Migration in U87 and T98G Cells

To explore whether Chalcone 9X could affect cell migration in glioma cells, Chalcone 9X was treated in human U87 and T98G for 48 h. Then, transwell assay and wound healing assay were performed to detect cell migration capacity. Results showed that Chalcone 9X treatment significantly repressed cell migration of U87 and T98G cells with dose dependency for 48 h (Figures 3(a)–3(d)) (*p* < 0.05). Furthermore, the wound healing assay also illustrated the inhibitory migration effect in U87 and T98G cells by Chalcone 9X treatment after 48 h (Figures 3(e)–3(h)) (*p* < 0.05). In addition, we detected some gene expressions of migration, such as Vimentin [22, 23], N-cadherin [24–26], and E-cadherin [27, 28]. Results showed that Chalcone 9X treatment repressed protein levels of Vimentin and N-cadherin and promoted E-cadherin expression with dose dependency in U87 and T98G cells after 48 h (Figures 3(i)–3(k)) (*p* < 0.05), which suggested that Chalcone 9X repressed cell migration in glioma cells. The above data indicated that Chalcone 9X could suppress cell proliferation and migration in glioma cells. However, the mechanism was not precise. Therefore, we intended to explore the potential mechanism of Chalcone 9X in treating glioma.

The article "Chalcone 9X Contributed to Repressing Glioma Cell Growth and Migration and Inducing Cell Apoptosis by Reducing FOXM1 Expression In Vitro and Repressing Tumor Growth In Vivo" was published in 2022. Journal: Biomed Res Int.

### 3.4. Chalcone 9X Repressed Protein Levels of FOXM1 in U87 and T98G Cells

In order to explore the mechanism, which Chalcone 9X regulated glioma cell proliferation and migration, we detected some signaling pathway molecules and oncogenes that played critical roles in cell proliferation and the development of glioma. Wnt/*β-*catenin and ERK/GSK3*β* signaling pathways were closely associated with cell proliferation and progression in glioma [29–35]. FOXM1 was an oncogene that could promote the development and malignancy of glioma [36–38]. Therefore, the protein levels of Wnt, *β*-catenin, p-*β*-catenin, ERK, p-ERK, GSK3*β*, p-GSK3*β*, and FOXM1 were detected by WB in U87 and T98G cells. Our results showed that no significant difference had been found in protein levels of Wnt/*β*-catenin, ERK/GSK3*β* signaling molecules (Figure 4) (*p* > 0.05). Results indicated that Chalcone 9X repressed the protein levels of FOXM1 in a dose-dependent manner in U87 and T98G cells after 48 h (Figure 4) (*p* < 0.05), which might suggest that Chalcone 9X might play some roles in glioma cell proliferation via the oncogenic factor FOXM1.

### 3.5. FOXM1 Overexpression Removed the Chalcone 9X Effects on Cell Proliferation, Apoptosis, and Migration in U87 and T98G Cells

To verify that Chalcone 9X repressed cell proliferation, migration, and induced cell apoptosis through repressing FOXM1 expression in glioma, the total length of FOXM1 was constructed into the plasmid, which was named p-FOXM1 and transfected into U87 and T98G cells. Then Chalcone 9X with 100 *μ*mol/L was added into the glioma cells with p-FOXM1 or p-NC for 48 h. The cell proliferation and migration capacities were observed. Results showed that the protein expressions of FOXM1 were upregulated after p-FOXM1 transfection into U87 and T98G cells, which suggested FOXM1 was successfully transfected into glioma cells, while FOXM1 protein levels were reduced after treating with Chalcone 9X (Figure 5(a)) (*p* < 0.001). Furthermore, the CCK-8 assay showed that the promoted cell viability in the p-FOXM1 group was repressed after treatment with Chalcone 9X (Figure 5(b)) (*p* < 0.001). Moreover, FACS assay showed that the reduced cell apoptotic rates in the p-FOXM1 group was increased after treating with Chalcone 9X (Figure 5(c)) (*p* < 0.001). Besides, the transwell assay illustrated that the promoted cell migration capacity in p-FOXM1 group was repressed after treating with Chalcone 9X (Figures 5(d) and 5(e)) (*p* < 0.001). In addition, the increased protein levels of Vimentin and N-cadherin and repressed protein levels of E-cadherin were reversed after treatment with Chalcone 9X in glioma cells (Figures 5(f)–5(h)) (*p* < 0.001). Above all, these data suggested that FOXM1 overexpression removed the Chalcone 9X effects on cell proliferation, apoptosis, and migration in U87 and T98G cells.

The article "Chalcone 9X Contributed to Repressing Glioma Cell Growth and Migration and Inducing Cell Apoptosis by Reducing FOXM1 Expression In Vitro and Repressing Tumor Growth In Vivo" was published in 2022. Journal: Biomed Res Int.

### 3.6. Chalcone 9X Inhibited U87 Tumor Growth of a Xenograft Model in Nude Mice

To verify the functions of Chalcone 9X, a xenograft tumor model of U87 cells in nude mice was used. After two weeks, Chalcone 9X with concentrations of 20 mg/kg and 40 mg/kg was treated in these nude mice for another four weeks. Then, these nude mice were sacrificed, and the tumor weight and tumor volumes were measured. Results showed that Chalcone 9X treatment could dramatically repress tumor weight and tumor volumes after treating for 21 d and 28 d in vivo, compared with the model group (Figures 6(a)–6(c)) (*p* < 0.01). Furthermore, upon increasing the Chalcone 9X dosage, the tumor weight and tumor volumes decreased, which indicated a dose-dependent manner in vivo (Figures 6(a)–6(c)) (*p* < 0.05). In addition, as previously introduced, the FOXM1-positive index is an oncogene for cancer development and a marker for cell proliferation [36–38], and the Caspase-3 is a marker for cell apoptosis [19]. As shown in Figure 6(d), the immunohistochemical analysis indicated that the FOXM1 indices of the 40 mg/kg and 20 mg/kg Chalcone 9X groups were remarkably suppressed in contrast to the untreated group. In comparison, the Caspase-3 indices of the 40 mg/kg and 20 mg/kg Chalcone 9X groups were improved in compared with the untreated group (Figures 6(d) and 6(e)) (*p* < 0.05). Besides, the WB assay showed that the protein levels of FOXM1, Vimentin, and N-cadherin were repressed, while E-cadherin was increased with dose dependency (Figures 6(f) and 6(g)) (*p* < 0.05), which indicated that the migrated capacity was also repressed in vivo. Collectively, these data suggested that Chalcone 9X could inhibit U87 tumor growth of a xenograft model in nude mice.

The article "Chalcone 9X Contributed to Repressing Glioma Cell Growth and Migration and Inducing Cell Apoptosis by Reducing FOXM1 Expression In Vitro and Repressing Tumor Growth In Vivo" was published in 2022. Journal: Biomed Res Int.

## 4. Discussion

Chalcones have been demonstrated to inhibit tumor progression and development in cancers [12–18], including glioma [15, 18]. The synthetic Chalcone 9X is an aromatic ketone, which has been proved to own antitumor activities in lung cancer cells and hepatic cancer cells through activating Caspase-3 and Caspase-8 signaling pathway [19]. The functions of Chalcone 9X in glioma cells remained unclear. In this study, we found that Chalcone 9X could suppress cell growth and induce cell apoptosis in glioma cells, and it showed little cytotoxicity to normal astrocyte cell line HA1800. As a result, we intended to explore the molecular mechanisms of Chalcone 9X in glioma cells.

In addition to its apoptotic and growth inhibitory functions, Chalcone 9X was also found to suppress the migration of glioma cells. N-cadherin and E-cadherin belong to the cadherin family, which have been found to regulate migration and metastasis in glioma [24–28]. Vimentin is a protein in the intermediate filament, which forms the cytoskeleton and is associated with cancer migration [22, 23]. We found that Chalcone 9X treatment inhibited cell migration and protein expressions of N-cadherin and Vimentin were repressed, while E-cadherin was increased, which confirmed that Chalcone 9X could repress migration in glioma cells, but the potential mechanisms remained unclear.

To explore the molecular mechanisms, we detected Wnt/*β-*catenin signal pathway [29–32], ERK/GSK3*β* pathway molecules [33–35], and P53 [39–41], which were associated with cell proliferation and progression in glioma [29–35, 39–41]. FOXM1 is a transcription factor of the Fox protein superfamily. It is upregulated in glioma, which acts as an oncogene to promote the progression and metastasis [36, 37, 42]. FOXM1 is known to promote invasion, angiogenesis, and progression of various cancer cells through induction of matrix metalloproteinase genes [38, 43]. For example, FOXM1 could elevate the MYBL2 level to promote the progression of human glioma [36]. Furthermore, FOXM1 could regulate glioblastoma cell proliferation and progression by modulating some cell cycle-related genes required for G1/S and G2/M^42^. In this study, we found that Chalcone 9X treatment repressed mRNA and protein expressions of FOXM1 in glioma cells after treating for 48 h, which suggested that Chalcone 9X might regulate cell proliferation and migration by reducing the oncogenic factor FOXM1 in glioma.

The article "Chalcone 9X Contributed to Repressing Glioma Cell Growth and Migration and Inducing Cell Apoptosis by Reducing FOXM1 Expression In Vitro and Repressing Tumor Growth In Vivo" was published in 2022. Journal: Biomed Res Int.

In addition, we found that FOXM1 overexpression blocked the effects of Chalcone 9X on cell proliferation, apoptosis, and migration in glioma cells. Finally, a xenograft tumor in vivo model of U87 cells in nude mice was used. Results proved that Chalcone 9X treatment could inhibit tumor growth and the tumor migrated protein expressions of N-cadherin and Vimentin in vivo. In this study, we found that Chalcone 9X showed a lower cytotoxic effect than Chalcones 1 for human normal cell lines, and the security is much better than Chalcones 1. 100 *μ*mol/L Chalcone 9X had little cytotoxicity to normal astrocyte HA1800 cells, while 100 *μ*mol/L Chalcone 1 showed very high cytotoxicity to nontumor cell line [15].

A report found that chalcone 9X could induce conformation changes of Caspase-3 protein into mature Caspase-3 or cleaved Caspase-3, which could induce cell apoptosis [19]. In this study, our data uncovered that chalcone 9X could repress cell proliferation and the migration and induce cell apoptosis, which is likely conferred by the ability of this compound to promote the activation of FOXM1, thereby downregulating N-cadherin and Vimentin expression, upregulating Caspase-3 and N-cadherin expression. Moreover, that might be a potential treatment for glioma.

## 5. Conclusion

In conclusion, this study showed that Chalcone 9X, a synthetic chemical chalcone, suppressed cell proliferation, the migration, and induced cell apoptosis in human glioma cells, and it has little cytotoxicity to normal astrocyte cells. Therefore, we uncovered a novel way that Chalcone 9X could inhibit FOXM1 expression and repress the progression and bio-functions of glioma cells, which might be a potential therapeutic drug for treating human glioma.

## Figures and Tables

**Figure 1:** Chalcone 9X suppressed cell proliferation in U87 and T98G cells. Chalcone 9X with various concentrations (0 *μ*mol/L, 20 *μ*mol/L, 50 *μ*mol/L, and 100 *μ*mol/L) was treated in human glioma cells (U87 and T98G) and human astrocyte cell line (HA1800) for 24 h, 48 h, and 72 h. (a–f) Cell viability were detected by CCK-8 assay after Chalcone 9X treatment in glioma cells. (g–i) Cell viability was detected by CCK-8 assay after Chalcone 9X treatment in HA1800 cells. ^∗^*p* < 0.05,  ^∗∗^*p* < 0.01, and^∗∗∗^*p* < 0.001.

**Figure 2:** Chalcone 9X induced cell apoptosis in U87 and T98G cells. Chalcone 9X (0 *μ*mol/L, 20 *μ*mol/L, 50 *μ*mol/L, and 100 *μ*mol/L) was treated in human glioma cells for 48 h. (a–d) Cell apoptotic rates were detected by FACS assay after Chalcone 9X treatment in glioma cells. ^∗^*p* < 0.05,  ^∗∗^*p* < 0.01, and^∗∗∗^*p* < 0.001.

The article "Chalcone 9X Contributed to Repressing Glioma Cell Growth and Migration and Inducing Cell Apoptosis by Reducing FOXM1 Expression In Vitro and Repressing Tumor Growth In Vivo" was published in 2022. Journal: Biomed Res Int.

**Figure 3:** Chalcone 9X repressed cell migration in U87 and T98G cells. Chalcone 9X (0 *μ*mol/L, 20 *μ*mol/L, 50 *μ*mol/L, and 100 *μ*mol/L) was treated into U87 and T98G cells for 48 h. (a–d) Transwell assay was used to detect cell migration capacity. (e–h) Wound healing assay was used to detect cell migration capacity. (i–k) Protein levels of Vimentin, N-cadherin, and E-cadherin were detected by WB assay (magnifications: ×1.5). ^∗^*p* < 0.05,  ^∗∗^*p* < 0.01, and^∗∗∗^*p* < 0.001.

**Figure 4:** Chalcone 9X repressed protein expressions of FOXM1 in U87 and T98G cells. Chalcone 9X (0 *μ*mol/L, 20 *μ*mol/L, 50 *μ*mol/L, and 100 *μ*mol/L) was treated in U87 and T98G cells for 48 h. (a–d) Protein expressions of Wnt, *β*-catenin, p-*β*-catenin, ERK, p-ERK, GSK3*β*, p-GSK3*β*, and FOXM1 were detected by WB in U87 and T98G cells (magnifications: ×1.5). ^∗^*p* < 0.05,  ^∗∗^*p* < 0.01, and^∗∗∗^*p* < 0.001.

**Figure 5:** FOXM1 overexpression removed the Chalcone 9X effects on cell proliferation, apoptosis, and migration in U87 and T98G cells. P-NC and p-FOXM1 were, respectively, glioma cells, and then 100 *μ*mol/L Chalcone 9X was treated in these cells for 48 h. (a) The mRNA levels of FOXM1 were detected by RT-PCR. (b) CCK8 assay was used to measure cell viability. (c) FACS assay was used to measure cell apoptosis. (d, e) Transwell assay was used to detect cell migration capacities. (f–h) The protein levels of Vimentin, N-cadherin, and E-cadherin in glioma cells were detected by WB (magnifications: ×0.8). ^∗∗^*p* < 0.01 and^∗∗∗^*p* < 0.001.

**Figure 6:** Chalcone 9X inhibited U87 tumor growth of a xenograft model in nude mice. U87 cells were injected into nude mice for two weeks; then Chalcone 9X (20 mg/kg, 40 mg/kg) was provided by gavage to these mice for another four weeks. (a) Images of 9 primary tumors at day 28 from the model group, Chalcone 9X 20 mg/kg group, and Chalcone 9X 40 mg/kg group after mouse scarification. (b) Tumor volumes were measured every seven days. (c) Tumor weights on day 28 after injection was calculated. (d, e) Immunohistochemical staining of FOXM1 and Caspase-3 in tumor tissue sections. (f, g) WB assay was performed to detect the protein expressions of FOXM1, Vimentin, N-cadherin, and E-cadherin. ^#^*p* < 0.05 and^###^*p* < 0.001, model group versus Chalcone 9X 20 mg/kg; ^∗∗∗^*p* < 0.001, model group versus Chalcone 9X 40 mg/kg.

## Data Availability

The datasets used and/or analyzed during the current study are available from the corresponding author on reasonable request.
